This article has been retracted.

# Combined effect of genetic background and gender in a mouse model of bleomycin-induced skin fibrosis

**DOI:** 10.1186/s13075-015-0659-5

**Published:** 2015-05-30

**Authors:** Nadira Ruzehaji, Jerome Avouac, Muriel Elhai, Maxime Frechet, Camelia Frantz, Barbara Ruiz, Joerg H. Distler, Yannick Allanore

**Affiliations:** INSERM U1016/UMR 8104, Cochin Institute, Paris, France; Rheumatology A Department, Paris Descartes University, Paris, France; Department of Internal Medicine and Institute for Clinical Immunology, University of Erlangen-Nuremberg, Erlangen, Germany; Institut Cochin, INSERM U1016, Bâtiment Gustave Roussy, 27 rue du Faubourg Saint Jacques 75014, Paris, France

## Abstract

**Introduction:**

Systemic sclerosis (SSc) is a connective tissue disorder characterised by the development of skin fibrosis. Our current understanding of the disease pathogenesis is incomplete and the study of SSc is hindered, at least partially, by a lack of animal models that fully replicate the complex state of human disease. Murine model of bleomycin-induced dermal fibrosis encapsulates important events that take place early in the disease course.

**Methods:**

To characterise the optimum *in vivo* parameters required for the successful induction of dermal fibrosis we subjected three commonly used mouse strains to repeated subcutaneous bleomycin injections. We aimed to identify the effects of genetic background and gender on the severity of skin fibrosis. We used male and female Balb/C, C57BL/6, and DBA/2 strains and assessed their susceptibility to bleomycin-induced fibrosis by measuring dermal thickness, hydroxyproline/collagen content and number of resident myofibroblasts, all of which are important indicators of the severity of skin fibrosis. All data are expressed as mean values ± SEM. The Mann–Whitney *U* test was used for statistical analysis with GraphPad Prism 6.04 software.

**Results:**

Dermal fibrosis was most severe in Balb/C mice compared to C57BL/6 and DBA/2 suggesting that Balb/C mice are more susceptible to bleomycin-induced fibrosis. Analysis of the effect of gender on the severity of fibrosis showed that male Balb/C, C57BL/6, DBA/2 mice had a tendency to develop more pronounced fibrosis phenotype than female mice. Of potential importance, male Balb/C mice developed the most severe fibrosis phenotype compared to male C57BL/6 and male DBA/2 as indicated by significantly increased number of dermal myofibroblasts.

**Conclusion:**

Our study highlights the importance of genetic background and gender in the induction of murine dermal fibrosis. Robust and reproducible animal models of fibrosis are important research tools used in pharmacological studies which may lead to better understanding of the pathogenesis of fibrotic diseases and assist in identification of new drugs.

## Introduction

Systemic sclerosis (SSc) is an autoimmune disorder characterised by progressive connective tissue fibrosis and life-threatening complications with high mortality and morbidity [1]. It has long been known that the level of available transforming growth factor-β (TGF-β), connective tissue growth factor and other profibrotic molecules in the dermis are critical for the development and sustaining of fibrosis in SSc [2]. Furthermore, dermal fibrosis in SSc is thought to be the result of activation and differentiation of fibroblasts into apoptosis-resistant and α-smooth muscle actin (α-SMA)-positive myofibroblasts. Increased expression of myofibroblasts further stimulates the formation of extracellular matrix (ECM) leading to aberrant skin architecture and pathological tissue remodelling [3]. There are no mechanistic-based therapies, such as pharmaceutical drugs, on the market that prevent and control the progression of excessive ECM formation in SSc. Thus, there is an urgent need to better understand fibrosis, devise processes for manipulating ECM formation and reduce excessive collagen deposition. The ability to develop novel anti-fibrotic therapies and analyse their efficacy in proof-of-concept (POC) studies is partly impeded by limitations in currently available animal models used to study this disorder in vivo. The pathophysiology of SSc is complex and believed to be caused by multiple factors including vasculopathy, inflammation, and autoimmunity [4, 5]. Not surprisingly, there is currently no animal model that perfectly mimics all the steps associated with the development of dermal fibrosis. Although there are several inducible and genetic models [4, 5], not a single one of these models recapitulates all of the clinical features consistent with human SSc [3]. The murine model of bleomycin-induced dermal fibrosis is widely used to study the changes that take place in the early phase of the disease [6]. Bleomycin is a glycopeptide-derived anti-tumor antibiotic, which was first isolated from a culture broth of *Streptomyces verticillus* [7]. Bleomycin induces the release of reactive oxygen species, recruitment of inflammatory cells, which activate resident fibroblasts and stimulate ECM formation. Due to its profibrotic properties, subcutaneous bleomycin is used to induce local skin fibrosis, which is known to persist for up to six weeks [8]. Apart from its local effect, high-dose subcutaneous bleomycin injections are thought to induce lung fibrosis [7] and systemic autoimmune responses characterised by the presence of antinuclear autoantibodies, such as anti-Scl-70, anti-U1 RNP [9].

The model of bleomycin-induced skin fibrosis, originally described by Yamamoto [10], has been used widely in preclinical [11] and pharmacological studies [12]. There are several modifications of this protocol, raising the issue of study-to-study variance of the resulting dermal fibrosis. Given that the bleomycin-induced model of SSc is an important tool in understanding the pathogenesis of fibrotic skin changes, we investigated the susceptibility and intensity of dermal fibrosis observed in mouse skin of three widely utilised mouse strains of both genders. We therefore hypothesised that different strains of mice will have various degrees of sensitivity in response to bleomycin-induced dermal fibrosis. The aim of this study was to suggest an optimised protocol and describe the methods necessary for the induction of a standardised model of fibrosis in adult mouse skin. The observations of this study are to be used as a guide to finding a suitable animal model, which is morphologically and histologically consistent with the early stages of SSc-associated skin fibrosis.

## Methods

### Murine model of bleomycin-induced dermal fibrosis

Three mouse stains, namely Balb/C, C57BL/6, DBA/2 (Janvier, Genest-St-Isle, France), were used in the studies. The Balb/C strain, originally created from a stock of outbred albino mice, was systematically inbred and has the following related genotype: Tyr^c^/ Tyr^c^, Tyrp1^b^/Tyrp1^b^, A /A - MHC: Haplotype H2^d^. The inbred strain of C57BL/6 mice (related genotype: a (a/a) non agouti - MHC: Haplotype H2^b^) is a widely used strain, which is frequently used as the genetic background in transgenic models. The DBA is the oldest of all inbred strains of mice, with the DBA/2 substrain having the following genotype: a/a, Tyrp1^b^/Tyrp1^b^, Myo5a^d^/Myo5a^d^ - MHC: Haplotype H2^d^.

To determine whether gender and mouse strain have an influence on the severity of dermal fibrosis we subjected one group of male Balb/C (n = 6), C57BL/6 (n = 6), and DBA/2 (n = 6) mice of 6 weeks of age, weighing 20–25 g, to bleomycin injections at a concentration of 0.5 mg/ml. The upper dorsa of mice were shaved and one square measuring 1 cm^2^ was drawn on the midline using a marker. We administered 100 μl of bleomycin (Laboratoire Roger Bellon, Neuilly-sur-Seine, France) at 0.5 mg/ml dissolved in PBS every other day for 21 days. As part of the protocol, bleomycin injection sites were rotated. The first four injections were administered into four different corners of the square followed by the fifth injection given in the middle of the square. This protocol was continued until the day of post-mortem examination, at which point the marked square created on the dorsal surface of mice was harvested, with one half of the biopsy specimen fixed in 4 % wt/vol. paraformaldehyde for histology and the other half snap frozen for molecular biology.

Another group of female Balb/C (n = 6), C57BL/6 (n = 6) and DBA/2 (n = 6) was subjected to bleomycin injections (100 μl of bleomycin at 0.5 mg/ml, every other day for 21 days). Age-matched control animals were treated with an equivalent dose of vehicle. Each experimental group consisted of 6 mice.

In a separated experiment, we aimed to assess whether the frequency of bleomycin injections had the capacity to alter the severity of dermal fibrosis. We subjected one group of male C57BL/6 mice (n = 6) of 6 weeks of age, weighing 20–25 g to bleomycin injections (0.5 mg/ml) given every day and another group (n = 6) to bleomycin injections (0.5 mg/ml) given every other day for 21 days. In a different experiment, we endeavoured to determine the effect of bleomycin dosage (C57BL/6 mice, bleomycin at 0.5 mg/ml vs 1 mg/ml administered every other day for 21 days) on the severity of dermal fibrosis. Mice were killed at 21 days after the first bleomycin experiment: 5 mm of lesional skin was harvested and fixed in 4 % wt/vol. buffered formalin and processed for histological analysis. Four lesional skin biopsies (3 mm each) were snap frozen in liquid nitrogen and used for colorimetric assessment of collagen content (hydroxyproline assay). All animal experiments were approved by the local Animal Ethics Committee (Comité National de Réflexion Ethique sur l’Expérimentation Animale-34) and principles of laboratory animal care were followed.

### Histology, immunohistochemistry and image analysis

Histological sections (4 μm) were cut from paraffin-embedded formalin-fixed lesional skin tissue. Sections were stained with haematoxylin and eosin (H&E) and images were captured at ×100 microscopic magnification. Histological dermal thickness was determined by manually drawing a straight line between the epidermis and adipose layer. Image analysis was performed using Image J software (a freely available Java image processing programme). Two independent assessors performed blinded measurements of histological slides.

We subjected 4 μm paraffin-embedded formalin-fixed samples of lesional skin to immunohistochemical analysis according to the manufacturer’s protocol (Dako, Carpinteria, CA, USA). Skin sections were deparaffinised, followed by antigen retrieval blocked in Super Block IDetect Super Stain System horseradish peroxidase (HRP) (ID Labs, London ON N4A 5 K2, Canada) for 10 minutes followed by incubation with 3 % H_2_O_2_ for 10 minutes to block endogenous peroxidase activity. Primary antibodies against α-SMA (1:500, Abcam, Cambridge, UK), CD3 (1:50, Abcam), CD22 (1:100, Abcam) and CD68 (1:100, Abcam) was applied overnight. Species-specific, biotinylated secondary antibodies (1:200) were used and detection was by Dako Liquid DAB Chromagen System (Dako). Myofibroblasts were identified by staining for α-SMA, as previously described [12]. The number of α-SMA-, CD3-, CD22- and CD68-positive cells was determined at high magnification in four different sections obtained from each mouse and determined by two blinded examiners. The number of α-SMA-, CD3-, CD22- and CD68-positive cells was counted and expressed as a number of total cells within each microscopic field normalised against NaCl control as previously described [12]. Negative controls included replacing primary antibodies with normal species-specific IgG.

### Assessment of inflammatory infiltrate

Assessment of the number of infiltrating mononuclear/inflammatory cells in bleomycin and NaCl-treated mouse skin was determined using H&E stained sections and immunohistochemical images of CD3-, CD22- and CD68-stained skin as described previously [12]. Eight different high-power fields from each mouse skin section were evaluated for inflammatory infiltrate by two independent examiners blinded to the treatment.

### Multiphoton microscopy

A multiphoton inverted stand Leica SP5 microscope (Leica Microsystems Gmbh, Wetzlar, Germany) was used for tissue imaging as previously described [13]. A Ti:Sapphire Chameleon Ultra (Coherent, Saclay, France) with a centre wavelength at 810 nm was used as the laser source for generating second harmonic generation (SHG) and two-photon excited fluorescence signals (TPEF). The laser beam was circularly polarized and we used a Leica Microsystems HCX IRAPO 25×/0.95 W objective. SHG and TPEF signals were detected in epi-collection through a 405/15-nm and a 525/50 bandpass filter, respectively, by NDD PMT detectors (Leica Microsystems) with a constant voltage supply, at constant laser excitation power, allowing direct comparison of SHG intensity values. LAS software (Leica, Germany) was used for laser scanning control and image acquisition.

### Masson’s trichrome staining

For direct visualisation of collagen fibres and histological assessment of collagen deposition, trichrome staining was performed using the Masson Trichrome Staining Kit (Sigma-Aldrich, St Louis, MO, USA). Skin sections stained with Masson Trichrome were visualised at ×200 microscopic magnification. All images were captured with Olympus BX63F microscope (Olympus, Tokyo, Japan) equipped with a digital signal processor CoolSNAP scientific CCD camera (Photometrics, Tucson, AZ, USA).

### Collagen measurements

The collagen content in lesional skin samples was explored by hydroxyproline assay. After digestion of punch biopsies (3 mm) in 6 M HCl for 3 hours at 120 °C, the pH of the samples was adjusted to 7 with 6 M NaOH. Samples were then mixed with 0.06 M chloramine T and incubated for 20 min at room temperature. Next, 3.15 M perchloric acid and 20 % p-dimethylaminobenzaldehyde were added and samples were incubated for additional 20 minutes at 60 °C. The absorbance was determined at 557 nm with a Spectra MAX 190 micro plate spectrophotometer (Molecular Devices, Sunnyvale, CA, USA).

### Statistics

All data are expressed as mean values ± standard error of the mean (SEM). The Mann-Whitney *U* test for non-related samples was used for statistical analysis with GraphPad Prism 6.04 software (San Diego, CA, USA). A *p* value of less than 0.05 was considered statistically significant.

## Results

### Pro-fibrotic effects of subcutaneous bleomycin injections in the dermis of male Balb/C, C57BL/6 and DBA/2 mice

To determine whether bleomycin had the same capacity to induce dermal fibrosis in three inbred mouse strains (Balb/C, C57BL/6 and DBA/2) that are frequently used for studies in dermal fibrosis research, we administered bleomycin at a concentration of 0.5 mg/ml, which was injected every other day for the period of 3 weeks. Assessment of dermal thickness, hydroxyproline content and myofibroblast count showed that bleomycin successfully induced dermal fibrosis in all of the three strains assessed (Fig. 1a-f). Bleomycin treatment in Balb/C, C57BL/6 and DBA/2 mice was associated with an increase in dermal thickness by 19.89 %, 21.31 % and 18.7 % respectively when compared to NaCl-treated counterparts (Fig. 1b). No significant difference in dermal thickness was found between bleomycin-treated male Balb/C, C57BL/6 and male DBA/2 mice (Fig. 1b). To confirm that the observed increase in dermal thickness in bleomycin-treated skin was due to increased collagen content, type I fibrillary collagen was imaged by SHG (Fig. 1c) and a hydroxyproline assay (Fig. 1d) was performed. Note similar baseline distribution of collagen fibre alignment in NaCl-treated Balb/C, C57BL/6 and DBA/2 mice (Fig. 1c, d). Consistent with increased dermal thickness in bleomycin treated groups, increased accumulation of collagen was observed in Balb/C, C57BL/6 and DBA/2 skin when compared to NaCl-treated controls (Fig. 1c; *p* = 0.0290 in Balb/C; *p* = 0.0001 in C57BL/6; *p* = 0.0103 in DBA/2).

**Fig. 1:** Histological and histochemical analysis of dermal fibrosis in male bleomycin-treated Balb/C, C57BL/6 and DBA/2 mice. **a** Representative images of H&E-stained sections of male mouse skin treated with subcutaneous NaCl or bleomycin given every other day over a period of 3 weeks. Original magnification ×100. **b** Dermal thickness of skin harvested from mice treated with NaCl or bleomycin after 3 weeks. Four high-power field images were taken (two measurements per image). Results represent the relative fold-change compared to NaCl-treated control mice. All values represent means ± standard error of the mean (SEM); n = 6 in each group. **c** Representative images of second harmonic generation imaging of type I fibrillary collagen in mouse skin harvested after 3 weeks of treatment with NaCl or bleomycin injected every other day. Note different distribution of fibre alignment and intensity in NaCl- and bleomycin-treated samples. Note that all images were acquired with the same excitation power. Original magnification ×250. **d** Hydroxyproline assay: results are represented as means ± SEM of triplicate measurements obtained from six mice (two biopsies per mouse) and shown as relative fold-change compared to NaCl-treated control samples. **e** Representative images of alpha smooth muscle actin (α-SMA) immunohistochemical analysis. Original magnification ×200, inset ×630. **f** Relative number of α-SMA-positive cells in the dermis of NaCl- or bleomycin-treated mice. Results represent the relative fold-change compared to NaCl-treated control mice. All values represent means ± SEM; n = 6 each group. *n.s*. not significant

Increased levels of collagen content in bleomycin-treated skin may result from increased recruitment of myofibroblasts. In order to determine whether myofibroblasts contributed to increased levels of collagen in the dermis of male Balb/C, C57BL/6 and DBA/2 mouse skin, we analysed the number of myofibrolbasts (Fig 1e-f). Under fibrotic conditions myofibroblast count increased five-fold in male Balb/C compared to NaCl control mice, two-fold in male C57BL/6 mice and three-fold in male DBA/2 mice. Male Balb/C mice treated with bleomycin had significantly increased dermal myofibroblast counts compared to bleomycin-treated male C57BL/6 mice (*p* = 0.0041) and DBA/2 mice (*p* = 0.05) (Fig 1f).

### Female Balb/C mice are more susceptible to bleomycin-induced dermal fibrosis than female C57BL/6 and DBA/2 counterparts

Dermal fibrosis was induced in female Balb/C, C57BL/6 and DBA/2 mice by subcutaneous bleomycin injections given for 3 weeks at a final concentration of 0.5 mg/kg and given every other day. Histological changes were determined by measuring dermal thickness in bleomycin-treated and NaCl control female Balb/C, C57BL/6 and DBA/2 mice. Dermal thickness was determined by measuring the average thickness between the epidermal–dermal and dermal–subcutaneous fat junctions.

Bleomycin treatment resulted in increased dermal thickness in female Balb/C mice compared to NaCl-treated female Balb/C mice (Fig. 2b; *p* = 0.0001). No significant difference was observed in dermal thickness in bleomycin-treated female C57BL/6 mice compared to NaCl-treated female controls (Fig. 2b), however, there was a 43.7 % increase (*p* = 0.0036) in collagen content and a 33.8 % increase (*p* = 0.0136) in myofibroblast count in female C57BL/6 mice compared to NaCl-treated female controls (Fig. 2c-d). There was no significant change in dermal thickness, hydroxyproline content or myofibroblast count in female DBA/2 mice treated with bleomycin compared to female DBA/2 mice treated with NaCl (Fig. 2a-f).

**Fig. 2:** Female Balb/C mice are more susceptible to bleomycin-induced dermal fibrosis than female C57BL/6 and DBA/2 mice. **a** Representative images of H&E-stained sections of female mouse skin treated with subcutaneous NaCl or bleomycin injections given every other day over a period of 3 weeks. Original magnification ×100. **b** Dermal thickness of skin harvested from female mice treated with NaCl or bleomycin after 3 weeks. Four high-power field images were taken (two measurements per image). Results represent the relative fold-change compared to NaCl-treated control mice. **c** Representative images of second harmonic generation imaging of type I fibrillary collagen in mouse skin harvested after 3 weeks of treatment with NaCl or bleomycin injected every other day. Original magnification ×250. **d** Hydroxyproline assay: results are represented as means ± standard error of the mean (SEM) of triplicate measurements obtained from six mice (two biopsies per mouse) and shown as relative fold-change compared to NaCl-treated control samples. **e** Representative images of α-SMA immunohistochemistry. Original magnification ×200, inset ×630. **f** Relative number of alpha smooth muscle actin (α-SMA)-positive cells in the dermis of NaCl- or bleomycin-treated mice. Results represent the relative fold-change compared to NaCl-treated control mice. All values represent means ± SEM; n = 6 in each group. *n.s*. not significant

### Effect of gender on the induction of experimental dermal fibrosis

To study the effect of gender on the induction of dermal fibrosis we compared fibrotic phenotype as determined by three parameters: dermal thickness, hydroxyproline content and myofibroblast count. Although male Balb/C and male C57BL/6 mice have scored higher in histological and immunohistochemical analysis of bleomycin-treated skin, there was no significant difference in dermal thickness, hydroxyproline and myofibroblast count between male and female Balb/C and C57BL/6 mice (Fig. 3a-c). The number of myofibroblasts in male DBA/2 mice was significantly higher than in female DBA/2 mice (Fig. 3c; *p* = 0.0355).

**Fig. 3:** Gender affects the severity of dermal fibrosis and inflammatory response. **a** Bleomycin-treated male Balb/C and male DBA/2 mice have slightly greater dermal thickness and **b** hydroxyproline content, compared to their female counterparts, however, this was not statistically significant. **c** Bleomycin-treated male DBA/2 mice have significantly higher myofibroblasts than their female counterparts. **d** Representative images of H&E-stained sections of male Balb/C, C57BL/6 and DBA/2 skin subjected to bleomycin (0.5 mg/ml) injections given every other day. **e** Relative number of inflammatory cells in the dermis of male Balb/C, C57BL/6 and DBA/2 mice in response to bleomycin injections. **f** Representative images of H&E-stained sections of skin subjected to bleomycin (0.5 mg/ml) injections given every other day in female Balb/C, C57BL/6 and DBA/2 mice. **g** Relative number of inflammatory cells in the dermis of female Balb/C, C57BL/6 and DBA/2 mice in response to bleomycin injections. Original magnification ×630. All values represent means ± standard error of the mean; n = 6 in each group. *n.s.* not significant

### Male DBA/2 mice have the lowest number of infiltrating leukocytes

In addition to fibrotic skin changes, repetitive bleomycin injections are known to cause skin inflammation as defined by increased number of leukocytes recruited to the lesional area [7]. To determine whether the type of mouse strain had an effect on the number of inflammatory cells and the rate of inflammation in bleomycin-treated skin (0.5 mg/ml, alternate days, 3 weeks), skin from male and female Balb/C, C57BL/6 and DBA/2 mice was stained with H&E and the number of leukocytes was counted (Fig. 3d, e). The number of leukocytes in skin from bleomycin-treated male Balb/C and C57BL/6 mice was 2.1 and 2.5-fold higher respectively than in bleomycin-treated male DBA/2 mice (Fig. 3d, e; *p* = 0.0142 and *p* = 0.0018, respectively). The type of mouse strain did not have an effect on the rate of inflammation in female mice as there was no significant difference in the number of leukocytes between female Balb/C, female C57BL/6 or female DBA/2 mice (Fig. 3e, g).

To identify the nature of infiltrating leucocytes and determine the influence of mouse strain on leucocyte infiltration, we next quantified the number of CD3-, CD22- and CD68-positive cells skin from male and female Balb/C, C57BL/6 and DBA/2 mice. The number of CD3-, CD22- and CD68-positive cells were significantly reduced in male DBA/2 bleomycin-treated skin compared to bleomycin-treated skin in male Balb/C and C57BL/6 mice (Fig. 4a-f). There appeared to be no difference between the number of CD3-, CD22- and CD68-positive cells in skin from bleomycin-challenged female Balb/C, C57BL/6 and DBA/2 mice (Fig. 4g-l).

**Fig. 4:** Male DBA-2 mice had reduced numbers of CD3, CD22 and CD68 cell infiltration into bleomycin-challenged mouse skin. Representative images of **a** CD3, **b** CD22 and **c** CD68 immunohistochemical analysis sections of skin from male Balb/C, C57BL/6 and DBA/2 mice subjected to bleomycin (0.5 mg/ml) injections given every other day. **d**-**f** Relative number of CD3-, CD22- and CD68-positive cells in the dermis of male Balb/C, C57BL/6 and DBA/2mice in response to bleomycin injections. Original magnification ×400. All values represent means ± standard error of the mean (SEM); n = 6 in each group. Representative images of **g** CD3, **h** CD22 and **i** CD68 immunohistochemical analysis sections of skin from female Balb/C, C57BL/6 and DBA/2 mice subjected to bleomycin (0.5 mg/ml) injections given every other day. **j-l** Relative number of CD3-, CD22- and CD68-positive cells in the dermis of female Balb/C, C57BL/6 and DBA/2 mice in response to bleomycin injections. Original magnification ×400. All values represent means ± SEM; n = 6 in each group

### Effect of frequency of bleomycin administration on the severity of mouse skin fibrosis

To establish whether the frequency of bleomycin injections had an effect on the severity of skin fibrosis, male C57BL/6 mice were given daily subcutaneous injections of bleomycin (at 0.5 mg/ml, 3 weeks) and compared to male C57BL/6 mice which were given bleomycin injections on alternate days (at 0.5 mg/ml, 3 weeks). In response to bleomycin, which was given either daily or on alternate days, dermal thickness increased in bleomycin-treated mice compared to NaCl-treated controls (Fig. 5a, b). Although there was no difference in dermal thickness between mice treated with bleomycin daily or on alternate days (Fig. 5b), collagen accumulation as determined by hydroxyproline content (Fig. 5d, *p* = 0.0173) was significantly elevated in mice treated with bleomycin on alternate days compared to those treated every day. While myofibroblast count was slightly higher in mice treated with bleomycin on alternate days compared to those treated every day, this was not statistically significant (Fig. 5f).

**Fig. 5:** Male C57BL/6 mice subjected to bleomycin injections on alternate days show higher dermal collagen content than male C57BL/6 mice given daily bleomycin injections. **a** Representative images of H&E-stained sections of male C57BL/6 mouse skin treated with subcutaneous NaCl or bleomycin injections given either daily or every other day over a period of 3 weeks. Original magnification ×100. **b** Dermal thickness of male C57BL/6 mouse skin treated with subcutaneous NaCl or bleomycin injections given either daily or every other day over a period of 3 weeks. Four high-power field images were taken (two measurements per image). Results represent the relative fold-change compared to NaCl-treated control mice. **c** Representative images of Masson’s Trichrome-stained sections of mouse skin harvested after 3 weeks of treatment with NaCl or bleomycin injected either every day or every other day. Original magnification ×100. **d** Hydroxyproline assay which was used as an indicator of collagen content in mouse skin treated with bleomycin every day vs alternate days. Results are represented as means ± standard error of the mean (SEM) of triplicate measurements obtained from six mice (two biopsies per mouse) and shown as relative fold-change compared to NaCl-treated control samples. **e** Representative images of alpha smooth muscle actin (α-SMA) immunohistochemical analysis. Original magnification ×200, inset ×630. **f** Relative number of α-SMA-positive cells in the dermis of mice treated with NaCl or bleomycin either every day or alternate days. Results represent the relative fold-change compared to NaCl-treated control mice. All values represent means ± SEM; n = 6 in each group

### Increasing bleomycin concentration from 0.5 mg/ml to 1 mg/ml does not increase collagen deposition and myofibroblast accumulation in dermal fibrosis

Male C57BL/6 mice were given subcutaneous injections of bleomycin at a final concentration of 0.5 mg/ml or 1 mg/ml (alternate days, 3 weeks). Increasing bleomycin concentration from 0.5 mg/ml or 1 mg/ml did not have an effect on the severity of dermal fibrosis. There was no difference in dermal thickness (Fig. 6a, b), hydroxyproline content (Fig. 6c, d) or myofibroblast count (Fig. 6e, f) in skin from mice injected with bleomycin at 0.5 mg/ml compared to mice injected with 1 mg/ml bleomycin.

**Fig. 6:** The effect of low (0.5 mg/ml) and high (1 mg/ml) doses of subcutaneous bleomycin injections on dermal thickness, collagen content and number of myofibroblasts in the skin of male C57BL/6 mice subjected to bleomycin on alternate days for 3 weeks. **a** Representative images of H&E-stained sections of male C57BL/6 mouse skin treated with subcutaneous NaCl or bleomycin injections (0.5 mg/ml or 1 mg/ml) given every other day for 3 weeks. Original magnification ×100. **b** Dermal thickness of male C57BL/6 mouse skin treated with subcutaneous NaCl or bleomycin injections (0.5 mg/ml or 1 mg/ml) given every other day for 3 weeks. Four high-power field images were taken (two measurements per image). Results represent the relative fold-change compared to NaCl-treated control mice. **c** Representative images of Masson’s Trichrome-stained sections of mouse skin harvested after 3 weeks of treatment with NaCl or bleomycin injections (0.5 mg/ml or 1 mg/ml) given every other day for 3 weeks. Original magnification ×100. **d** Hydroxyproline content in skin treated with low or high (0.5 mg/ml or 1 mg/ml) doses of bleomycin. Results are represented as means ± standard error of the mean (SEM) of triplicate measurements obtained from six mice (two biopsies per mouse) and shown as relative fold-change compared to NaCl-treated control samples. **e** Representative images of alpha smooth muscle actin (α-SMA) immunohistochemical analysis in skin from mice treated with subcutaneous NaCl or bleomycin injections (0.5 mg/ml or 1 mg/ml) given every other day for 3 weeks. Original magnification ×200, inset ×630. **f** Relative number of α-SMA-positive cells in the dermis of mice treated with NaCl or bleomycin (0.5 mg/ml vs 1 mg/ml) on alternate days. Results represent the relative fold-change compared to NaCl-treated control mice. All values represent means ± SEM; n = 6 in each group

## Discussion

Bleomycin-treated Balb/C mice have the most severe fibrosis phenotype compared to C57BL/6 and DBA/2 mice, suggesting that the severity of skin fibrosis, apart from other factors such as the route of administration and dose of bleomycin [14], also depends on the genetic background of mice. Male Balb/C mice had a greater number of myofibroblasts than C57BL/6 and DBA/2 mice of the same gender. Female Balb/C mice were previously shown to have higher susceptibility to bleomycin with greater dermal thickness than their female C57BL/6 and DBA/2 counterparts [14]. Similarly, in this study female Balb/C mice had greater levels of skin fibrosis characterised by increased dermal thickness, greater deposition of collagen and elevated number of dermal myofibroblasts, suggesting that Balb/C mice (at least the female Balb/C mice mice), may be more susceptible to bleomycin-induced skin fibrosis than their C57BL/6 and DBA/2 counterparts.

To determine the effect of gender on the severity of skin fibrosis, Balb/C, C57BL/6 and DBA/2 mice of both genders were used to induce and assess the extent of fibrosis. Male mice tended to have a more pronounced fibrosis phenotype than female mice and, as observed in DBA/2 mice, had significantly elevated numbers of myofibroblasts than female C57BL/6 and DBA/2 mice.

The fact that male mice are more susceptible to the development of SSc-associated skin fibrosis is in agreement with epidemiological observations, which suggest that although women have greater susceptibility to SSc than men, male patients are known to have a more severe skin fibrosis phenotype [3, 15]. Age is another factor that may have impacted on our study. Human studies indicate that most women are diagnosed with SSc later in life and generally after the onset of menopause [16], whereas animals used in the current study were young and sexually active mice of both genders. Therefore, differences in the severity of fibrosis observed between the genders were possibly due to age, which in turn is characterised by differential expression of sex hormones. For instance, oestrogen was previously shown to have an influence on the development of SSc-associated fibrosis [17] with low levels of oestrogen being associated with severe fibrosis and exacerbated pulmonary hypertension [17]. Oestrogen levels are at their lowest after the menopause and highest during pregnancy. Given that most women are diagnosed with SSc at the time when their oestrogen levels are at their lowest [16], and some autoimmune diseases, including rheumatoid arthritis [18], go into remission when oestrogens are at their peak, suggests that oestrogen may play an important protective role in autoimmune diseases such as SSc. Consistent with the observations in human SSc, increased circulating levels of oestrogen in young female compared to young male mice may have had a protective effect against the development of fibrosis, offering a plausible explanation as to why male mice developed a more severe fibrosis phenotype than female mice.

Studying the characteristics of skin changes that develop as a result of repetitive bleomycin injections [10] can help us to better understand inflammation and fibrosis, both of which are key elements that recapitulate pathological events in SSc. Increased inflammatory infiltrate in lesional skin in SSc, predominantly CD4+ T cells [19], suggests a distinct role of CD4 lymphocytes in the development of skin fibrosis. In animal experiments, bleomycin evokes a proinflammatory response and increased prevalence of leukocytes. Due to its complexity and the involvement of multiple organs, SSc is difficult to replicate in vivo. While many animal models of SSc exist [4] there is currently no animal model that can capture this complexity. Along with its disadvantages, namely the absence of vascular complications [5], the bleomycin-induced model of skin fibrosis provides us with an opportunity to study inflammation, elucidate the pathophysiology of SSc and explore potential treatment interventions. Inflammatory cells are thought to contribute to the initial activation of resident fibroblasts by the release of profibrotic mediators. To assess the contribution of genetic background on the development of inflammation associated with dermal fibrosis, Balb/C, C57BL/6 and DBA/2 mice of both genders were treated for 3 weeks with subcutaneous injections of bleomycin. Given that male DBA/2 mice had the least number of CD3-, CD22- and CD68-positive inflammatory cells, we suggest that in studies focusing on investigating the effect of inflammation on the pathogenesis of dermal fibrosis, strains other than DBA/2 are used. The number of inflammatory cells in bleomycin-treated male C57BL/6 mice was three times higher than the number of leucocytes found in DBA/2 mice, suggesting that C57BL/6 could be a strain of choice in studies of inflammation.

Having established the fact that male mice are more susceptible to dermal fibrosis than female mice we used male C57BL/6 mice to investigate whether varying the frequency of bleomycin injections (every day versus alternate days) affects the severity of dermal fibrosis. Bleomycin stimulates extracellular matrix formation by virtue of its profibrotic effects, and importantly, our studies indicated that daily exposure to bleomycin blunted the pro-fibrotic response of bleomycin in the skin, whereas alternate-day administration enhanced this effect. Bleomycin injections administered on alternate days resulted in increased basal hydroxyproline, a biochemical marker of collagen, compared to daily injections. Local bleomycin injections are associated with active stimulation of leukocyte infiltration [20] driving the release of a plethora of proinflammatory cytokines including TGF-β1, which in turn promotes the synthesis and secretion of collagen and other matrix molecules [21]. Enhanced immune response and consequent TGF-β activation aggravates fibrosis, as it sets up a positive feedback, which could partially explain why bleomycin injections given on alternate days are more efficient in stimulating the extracellular matrix. Alternate-day injections may cause peaks of cytokine release in the skin and stimulate a more sustained inflammatory response than bleomycin injections given daily. The frequent peaks of proinflammatory cytokine release induced by bleomycin injections administered on alternate days versus daily injections might be important in mediating an efficient profibrotic effect of bleomycin. Bleomycin increased skin collagen levels in a dose-dependent manner and, although doses ≤0.5 mg/ml are reported to induce histological changes [10], our studies suggest that fibrotic responses are similar in mice treated with low (0.5 mg/ml) and high (1 mg/ml) doses of bleomycin.

## Conclusions

In this study we evaluated the potential for the genetic background and gender of mice to effect the induction of experimental mouse dermal fibrosis. With the information present herein, we suggest that dermal fibrosis studies are best done in male rather than female mice due to higher responsiveness to bleomycin injections. Optimum results are obtained using the C57BL/6 strain by treating the mice with subcutaneous bleomycin at a final concentration of 0.5 mg/ml administered on alternate days. These observations are of considerable importance in the selection of an appropriate protocol for the induction of dermal fibrosis, which may be used in pharmacological testing and therapeutic interventions.

## Abbreviations

ECM: extracellular matrix
H&E: haematoxylin and eosin
HRP: horseradish peroxidase
PBS: phosphate-buffered saline
SHG: second harmonic generation
SSc: systemic sclerosis
TGF-β: transforming growth factor beta
α-SMA: alpha smooth muscle actin
